The article "The Efficacy and Safety of Bisoprolol in the Treatment of Myocardial Infarction with Cardiac Insufficiency" was retracted in 2023. Reasons: unreliable results or conclusions; concerns about the data; concerns about the peer review; concerns about the citations.

# The Efficacy and Safety of Bisoprolol in the Treatment of Myocardial Infarction with Cardiac Insufficiency

**DOI:** 10.1155/2022/3098726

**Published:** 2022-08-25

**Authors:** Yan Wang

**Affiliations:** Sixth Department of Cardiology, Cangzhou Central Hospital, Cangzhou, 061000 Hebei Province, China

## Abstract

**Background:**

Bisoprolol is commonly used to treat moderate or severe chronic stable heart failure, coronary heart disease, and hypertension. This study is aimed at analyzing the efficacy of bisoprolol in the treatment of myocardial infarction with cardiac insufficiency and its effect on cardiac function, Hcy, and CRP through meta-analysis.

**Methods:**

A total of 120 patients with myocardial infarction and cardiac insufficiency from February 2020 to February 2021 were selected and randomly divided into two groups (control and the observation, *n* = 60) according to the random number table method. The control group was given conventional treatment. The observation group was given bisoprolol on the basis of control group. The clinical efficacy, systolic blood pressure, diastolic blood pressure, heart rate, cardiac function indexes, homocysteine (Hcy), and C-reactive protein (CRP) levels were compared between the two groups before and after treatment through data analysis. Adverse reactions were observed during treatment.

**Results:**

Compared with the control group, the total effective rate of the observation group was significantly increased (*p* < 0.05). After treatment, the levels of heart rate, left ventricular end-diastolic volume (LVEDV), and left ventricular end-systolic volume (LVESV) and serum Hcy and CRP levels in the observation group were significantly lower than those in the control group (*p* < 0.05). Meanwhile, left ventricular ejection fraction (LVEF) level in the observation group after treatment was higher than that of the control group (*p* < 0.05).

**Conclusion:**

Bisoprolol combined with conventional treatment can reduce serum Hcy and CRP levels in patients with myocardial infarction and cardiac insufficiency and improve cardiac function. Moreover, there are no obvious adverse reactions during the treatment.

## 1. Introduction

Myocardial infarction refers to acute myocardial ischemia and necrosis. Most myocardial infarctions result from severe and persistent acute ischemia of the corresponding myocardium due to a dramatic reduction or interruption of coronary blood supply. [1]. At present, the incidence of acute myocardial infarction in China is on the rise, and the incidence in rural areas is higher than that in urban areas. The mortality rate of myocardial infarction is on the rise [2, 3]. Cardiac insufficiency is a symptom of a decrease in myocardial contractile function, which reduces the forward blood flow of the heart, resulting in blood stasis in the systemic or pulmonary circulation [4, 5]. Previous studies have shown that after myocardial infarction, a large number of patients can induce or even aggravate cardiac insufficiency due to the greater impact of myocardial remodeling on cardiac contractility [6]. Myocardial infarction with cardiac insufficiency undoubtedly increases the difficulty of treatment and threatens the prognosis of patients.

Many studies have shown that patients with myocardial infarction and cardiac insufficiency cannot obtain reliable efficacy with conventional medical methods alone [7, 8]. Bisoprolol is a beta1-adrenoceptor blocker, which is commonly used in the treatment of moderate or severe chronic stable heart failure, coronary heart disease, and hypertension [9–11]. Bisoprolol is a widely used beta-blocker, whose primary mechanism is to block the connection between adrenaline and beta1 receptors [12]. Bisoprolol is more selective for *β*1 receptors than metoprolol and attilol. In addition, reliable efficacy has been achieved in the treatment of congestive heart failure [13, 14]. However, the effect of bisoprolol on myocardial infarction and cardiac insufficiency is unclear.

Therefore, this study tried bisoprolol and conventional treatment to treat patients with myocardial infarction and cardiac insufficiency. The efficacy of bisoprolol for myocardial infarction with cardiac insufficiency and its effects on cardiac function, Hcy, and CRP through meta-analysis were analyzed. This study will provide a reference for clinical treatment of patients with myocardial infarction and cardiac insufficiency.

## 2. Materials and Methods

### 2.1. Patients

This is a retrospective study. A total of 120 patients with myocardial infarction and cardiac insufficiency in Cangzhou Central Hospital from February 2020 to February 2021 were randomly divided into two groups according to the random number table method. This study was approved by the Ethics Committee of Cangzhou Central Hospital. The control group included 34 males and 26 females. The age of the patients ranged from 42 to 71 years, with an average of (57.25 ± 4.11) years. NYHA classification of cardiac function showed that the control group included 35 cases at grade II and 25 cases at grade III. The observation group included 36 males and 24 females. The ages of these patients ranged from 44 to 70 years old, with an average of (57.66 ± 4.23) years. NYHA classification of cardiac function showed that the observation group included 38 cases at grade II and 22 cases at grade III. There was no significant difference in general data between the two groups, and they were comparable.

### 2.2. Inclusion and Exclusion Criteria

Inclusion criteria: all patients signed informed consent. All patients received clinical symptoms, signs, and imaging diagnosis in Cangzhou Central Hospital. The diagnosis was made based on the diagnostic criteria in the “Guidelines for Primary Diagnosis and Treatment of ST-Segment Elevation Myocardial Infarction (2019)”. Patients were divided into grades II to III according to the New York Heart Association (NYHA) cardiac function classification. Patients were 60 years of age and older.

Exclusion criteria: patients with other system and organ dysfunction; patients with a history of drug allergy in this study; patients with severe heart failure; and patients with missing clinical data.

### 2.3. Treatment

The control group was given conventional treatment. After admission, the patients were given basic oxygen inhalation treatment and ECG monitoring. At the same time, cardiac, analgesic, and vasodilator treatments were given according to the patient's condition. The patients were given oral aspirin (Hunan Zhongnan Pharmaceutical Co., Ltd., Chinese medicine H43021055), nitroprom (China Resources Shuanghe Pharmaceutical Co., Ltd., Chinese medicine H11020907), nitroglycerin (Beijing Yimin Pharmaceutical Co., Ltd., Chinese medicine H11020289), and other drugs. Antiarrhythmic therapy was used in patients with cardiac arrhythmias. For patients with dyspnea, furosemide and diuresis were given. The observation group was given bisoprolol (Beijing Huasu Pharmaceutical Co., Ltd., H10970082) and conventional treatment. The initial dose of bisoprolol was 6.25 mg twice a day. The dosage of bisoprolol is adjusted according to the patient's heart rate and blood pressure. The frequency of drug dose adjustment was 3 to 5 days, and the dose was adjusted to 12.5 mg. Then, the drug dose was gradually increased (25 mg/d ≤ drug dose ≤ 50 mg/d). All patients were treated continuously for 6 months.

### 2.4. Efficacy Evaluation Criteria

Markedly effective: after treatment, the patient's cardiac function improved by more than 2 grades, and the clinical symptoms and signs disappeared.

Effective: after treatment, patient's cardiac function improved to grade 2 or above, and the clinical symptoms and signs improved.

Invalid: the patient's cardiac function, clinical symptoms, and signs did not improve or even worsened after treatment.

(1) $$\begin{array}{c} \text{Total effective}=\text{markedly effect}+\text{effective}. \end{array}$$

### 2.5. Observation Index

The levels of serum Hcy, CRP and clinical efficacy, systolic blood pressure, diastolic blood pressure, heart rate, and cardiac function indexes were compared between the two groups before and after treatment. Meanwhile, adverse reactions were monitored during treatment.

Left ventricular end-diastolic volume (LVEDV), left ventricular end-systolic volume (LVESV), and left ventricular ejection fraction (LVEF) were measured by Mindray DC-N3S color Doppler before and after treatment.

Fasting venous blood (5 ml) before and after treatment was put in a centrifuge and centrifuged at 2500 rpm for 10 min. The extracted serum was placed in the refrigerator for testing. CRP levels were measured using an enzyme-linked immunosorbent assay (ELISA). HCY levels were measured using an automatic immunoassay analyzer.

### 2.6. Statistical Analysis

All experiments were performed in triplicate. Data were analyzed using SPSS18.0 statistical software. Differences between groups were compared using *χ*^2^ test and *t* test. Count data were expressed as %, and measurement data were expressed as mean ± SD. *p* < 0.05 represented statistical significance.

## 3. Results

### 3.1. Comparison of Clinical Efficacy between the Two Groups

The observation group found a total of 53 effective people. The data showed that the total effective rate of the observation group was 88.33%. Meanwhile, 44 effective people were found in the control group. The total effective rate in the control group was 73.33%. Compared with the control group, the total effective rate of the observation group was significantly increased (*p* < 0.05, Table 1).

### 3.2. Comparison of Heart Rate, Systolic Blood Pressure, and Diastolic Blood Pressure between the Two Groups before and after Treatment

After treatment, the heart rate in both groups was significantly decreased. Compared with the control group, the heart rate of the observation group was significantly decreased (*p* < 0.01, Table 2). After treatment, there were no changes in systolic and diastolic blood pressure in the two groups (*p* > 0.05, Table 2). There were no significant changes in systolic and diastolic blood pressure between the two groups (*p* > 0.05, Table 2).

### 3.3. Comparison of Cardiac Function Indexes between the Two Groups before and after Treatment

After treatment, the levels of LVESV and LVEDV in the two groups were decreased, and the level of LVEF was increased. In addition, compared with the control group, the levels of LVESV and LVEDV in the observation group were significantly decreased, and the level of LVEF was significantly increased (*p* < 0.01, Table 3).

### 3.4. Comparison of Serum Hcy and CRP Levels between the Two Groups before and after Treatment

After treatment, serum Hcy and CRP levels in both groups were decreased. In addition, the serum Hcy and CRP levels in the observation group were lower than those in the control group (*p* < 0.01, Table 4). Moreover, there were no obvious adverse reactions during treatment in both groups.

## 4. Discussion

After myocardial infarction, the myocardium is prone to systolic and diastolic dysfunction, which induces and aggravates the occurrence and development of cardiac insufficiency, and even induces heart failure in severe cases [8, 15]. In the current clinical work, the treatment of myocardial infarction complicated with cardiac insufficiency mainly focuses on cardiotonic, diuretic, and coronary artery expansion [16, 17]. However, these medical treatments are more common. Moreover, long-term use of angiotensin-converting enzyme inhibitors in patients is very likely to induce the phenomenon of “aldosterone escape,” causing unnecessary damage to the heart [18–20]. The application of *β*-blockers can increase the density of *β*-receptors and have a strong antagonistic effect on catecholamines, thereby reducing cardiotoxicity and enhancing myocardial response [21].

Bisoprolol, as a specific *β*1 adrenergic receptor blocker, is commonly used in clinical practice and has the advantages of low first-pass effect and long half-life [22]. And bisoprolol is also highly absorbed orally and more easily crosses the blood-brain barrier. Bisoprolol not only has a strong blocking effect on part of *β*1 but also significantly reduces the possible adverse reactions to the central nervous system [23]. In addition, it was found that the application of bisoprolol can not only effectively reduce the heart rate but also have a strong inhibitory effect on the release of renin [24]. Bisoprolol can improve the hypoxic state of myocardium and also has a strong recovery effect on myocardial systolic and diastolic function. Therefore, bisoprolol can effectively reduce the scope of myocardial infarction and ultimately achieve the purpose of eliminating and relieving clinical symptoms and signs [25]. It has also been reported that early treatment with bisoprolol can reduce the incidence of arrhythmias to a certain extent [26]. The results showed that bisoprolol and conventional treatment improved cardiac function and reduced heart rate in patients. It indicates that the application of bisoprolol can not only produce a strong vasoconstriction effect but also help to reduce the excitability of sympathetic nerves. Bisoprolol prolongs ventricular diastolic filling time to a certain extent and reduces cardiac load [27]. Ultimately, bisoprolol improves myocardial compliance, increases coronary blood perfusion, and effectively improves clinical symptoms and signs in patients with myocardial infarction and cardiac insufficiency.

At the same time, serum Hcy and CRP levels were also observed in this study. Serum Hcy is considered a commonly used specific indicator for assessing cardiovascular disease outcomes [28]. CRP is a more sensitive indicator of human inflammatory response [29]. The results of this study show that bisoprolol can effectively regulate serum Hcy and CRP levels, further confirming the superiority of bisoprolol in the treatment of myocardial infarction with cardiac insufficiency. In addition, since bisoprolol is metabolized in the human body through the dual channels of liver and kidney [30], it does not cause serious adverse reactions. However, it should be noted that bisoprolol may cause mild to moderate renal and hepatic insufficiency [31]. In this study, no obvious adverse reactions were found in patients with myocardial infarction and cardiac insufficiency after treatment, indicating that the safety of bisoprolol is still high. In the following research, the sample size and observation indicators will be further increased to better evaluate the application advantages of bisoprolol.

## 5. Conclusion

Data analysis showed that bisoprolol combined with conventional treatment can effectively improve the heart rate and cardiac function in patients with myocardial infarction and cardiac insufficiency. At the same time, bisoprolol can regulate serum Hcy and CRP levels and do not have adverse reactions. Therefore, bisoprolol is a safe and effective drug for patients with myocardial infarction and cardiac insufficiency.

## Figures and Tables

**Table 1:** Comparison of clinical efficacy between the two groups [case (%)].

Group	Case	Markedly effective	Effective	Invalid	Total effective rate
Control	60	23 (38.33)	21 (35.00)	16 (26.67)	44 (73.33)
Observation	60	29 (48.33)	24 (40.00)	7 (11.67)	53 (88.33)
*χ* ^2^					4.357
*p*					0.037^∗^

^∗^ *p* < 0.05.

**Table 2:** Comparison of heart rate, systolic blood pressure, and diastolic blood pressure between the two groups before and after treatment.

Group	Heart rate (times/min)		Systolic blood pressure (mmHg)		Diastolic blood pressure (mmHg)	
	Before	After	Before	After	Before	After
Control	115.22 ± 3.6	98.33 ± 2.2	119.36 ± 21.2	118.60 ± 22.2	74.25 ± 15.4	74.11 ± 14.5
Observation	116.15 ± 4.1	75.65 ± 1.2	120.15 ± 22.1	119.31 ± 23.1	75.10 ± 14.2	72.60 ± 12.7
*t*	1.312	69.326	0.200	0.172	0.412	0.605
*p*	0.192	*p* ≤ 0.001^∗∗^	0.842	0.864	0.682	0.546

^∗∗^ *p* < 0.01.

**Table 3:** Comparison of cardiac function indexes between the two groups before and after treatment.

Group	LVESV (ml)		LVEDV (ml)		LVEF (%)	
	Before	After	Before	After	Before	After
Control	54.21 ± 12.5	50.98 ± 12.7	94.25 ± 16.5	92.68 ± 14.1	38.65 ± 2.55	48.65 ± 5.11
Observation	55.10 ± 11.6	44.83 ± 10.5	94.10 ± 15.8	86.11 ± 5.2	39.11 ± 2.76	54.10 ± 5.41
*t*	0.403	2.884	0.051	3.380	0.948	7.269
*p*	0.688	0.005^∗∗^	0.960	0.001^∗∗^	0.345	*p* ≤ 0.001^∗∗^

^∗∗^ *p* < 0.01.

**Table 4:** Comparison of serum Hcy and CRP levels before and after treatment in the two groups.

Group	Hcy (*μ*mol/l)		CRP (mg/l)	
	Before	After	Before	After
Control	19.25 ± 4.02	16.40 ± 2.81	21.45 ± 3.15	12.64 ± 2.47
Observation	19.31 ± 4.11	12.34 ± 3.20	22.50 ± 2.79	8.75 ± 1.24
*t*	0.081	7.385	1.933	10.902
*p*	0.936	*p* ≤ 0.001^∗∗^	0.056	*p* ≤ 0.001^∗∗^

^∗∗^ *p* < 0.01.

## Data Availability

The datasets used and/or analyzed during the present study are available from the corresponding author on reasonable request.
